# The Comparison of Clinical Efficacy of Minimally Invasive Tarsal Sinus Approach and L-Type Incision Approach Combined with 3D Printing Technology in Calcaneal Fracture

**DOI:** 10.1155/2022/5706341

**Published:** 2022-07-11

**Authors:** Hao Du, Shiang Li, Shicheng Tu, Kun Wang, Zhiyu Fang

**Affiliations:** The First Affiliated Hospital, and College of Clinical Medicine of Henan University of Science and Technology, Luoyang, China 471003

## Abstract

**Purpose:**

To explore the comparison of the reduction of the subtalar articular surface and other postoperative effects of the minimally invasive tarsal sinus approach and lateral L-shaped incision conventional approach for the treatment of calcaneal fracture with 3D printing technology.

**Methods:**

Patients who received surgical treatment for calcaneal fractures in the First Affiliated Hospital of Henan University of Science and Technology from June 2019 to December 2020 were collected. 3D printing equipment produced the affected side reduction heel bone fracture model and navigation template model. The tarsal sinus approach was used in the experimental group, and the lateral L-shaped incision approach was used in the control group. Patients were followed up 3 days, 1 month, 3 months, 6 months, and 12 months after the operation. Imaging indicators were measured 12 months after surgery, and scores from American Foot and Ankle Orthopaedic Society (AOFAS) and MSF were performed.

**Results:**

Operation time was 70.52 ± 13.16 in the control group and 55.24 ± 12.25 minutes in the experimental group (*P* < 0.001). Intraoperative blood loss was 98.77 ± 18.65 in the control group and 89.56 + 17.54 in the experimental group (*P* > 0.05). The duration of antibiotic use was 5.53 ± 3.24 days in the control group and 5.48 ± 4.18 days in the experimental group (*P* > 0.05). The frequency of fluoroscopy was 6.56 ± 1.72 in the control group and 3.88 ± 1.05 in the experimental group (*P* < 0.001). Fracture healing time was 3.24 ± 0.52 months in the control group and 3.08 ± 0.58 months in the experimental group (*P* > 0.05). The postoperative Böhler angle was 28.31 ± 3.14 in the control group and 29.24 ± 2.76 in the experimental group (*P* > 0.05). Postoperative subtalar articular displacement (step > 2 mm) was observed in 4 patients in the control group and 1 in the experimental group (*P* < 0.05). MSF score was 90.12 ± 4.85 in the control group and 91.36 ± 2.58 in the experimental group (*P* > 0.05).

**Conclusion:**

The study found that the experimental group was significantly better than the control group in terms of the operation time, intraoperative fluoroscopy times, and success rate of reduction of the subtalar articular surface. 3D printing technology can shorten the operation time, accurately reduce the fracture block, and reduce the secondary trauma, which is conducive to the functional recovery of the affected foot.

## 1. Introduction

Calcaneal fracture is a common fracture, accounting for about 2% of all fractures in the human body. Degloving of the sole of the foot is rare and serious since the heel pad cannot be replaced by a similar tissue [1]. It usually occurs after high-energy axial trauma, such as falling from a height or automobile accident, and brings huge economic and social burden to patients [2]. It typically takes 5-10 months for patients to return to work, with about 20% of patients unable to return to work within a year [3]. Retrocalcaneal articular surface involvement is considered to be the most predictable cause of severe adverse outcomes because of the increased likelihood of postoperative osteoarthritis and its attendant pain and chronic stiffness [4]. Open reduction and internal fixation have been the most common techniques over the past few decades, and it remains the standard treatment of choice [5]. Usually through a lateral approach, wound infection and rupture and flap loss and sural nerve injury are associated [6]. The management of displaced intra-articular calcaneal fractures (DIACF) is a challenging task due to the irregular anatomy of the calcaneus, its complex coupling with the talus, and its fragile soft tissue capsule [7–9].

In order to maintain the normal function of the subtalar joint and hindfoot and reduce the incidence of complications, accurate and personalized surgery is becoming increasingly important in fracture fixation. When the patient is symptomatic, an optimal functional outcome can only be obtained after operative treatment. There is currently no consensus on the best surgical technique to treat this condition [10]. Preoperative 3D modeling can diagnose and simulate the surgical process more effectively [11]. 3D printing technology, also known as additive manufacturing and rapid prototyping, has emerged in the past 30 years, providing a variety of applications in clinical practice, highlighting preoperative planning, simulation of surgical strategies, and teaching and communication between orthopedic and reconstructive surgery and patients [12].

People use this technology to make 3D physical models, carry out surgical planning, simulate the surgical process, establish surgical guidance templates, and design personalized internal plants or artificial joint prostheses [13]. 3D models can be used to observe intra-articular calcaneal fractures, especially the fracture displacement of calcaneocuboid and subtalar surfaces [14]. It is more intuitive to show the internal calcaneal fractures such as the splitting of medial loading talus process, separation of calcaneal tubercle, colliculus collapse, and lateral burst bone. The hook plate technique is a strong fixation method for fracture-avulsion, raising the possibility of earlier joint movements and rapid recovery [15]. We assist surgeons to formulate and optimize surgical procedures before surgery and simulate and practice the surgical process, thus shortening the operation time.

This study applied 3D printing technology and remodel patients' calcaneal fracture block to evaluate its feasibility, accuracy, and predictability in fracture repair surgical planning. It mainly demonstrated the application of 3D printing technology in osteology and will provide important real evidence for surgeons. The aim was to diagnose correctly and make individualized surgical plans, to improve the safety and effectiveness of surgery significantly.

## 2. Methods

### 2.1. Research Subjects

Patients with calcaneal fractures who received surgical treatment in the Department of Orthopedics of the First Affiliated Hospital of Henan University of Science and Technology from June 2019 to December 2020 were included in the study. Patients were divided into experimental groups and control groups according to the choice of operation methods. The tarsal sinus approach was used in the experimental group, and the lateral L-shaped incision approach was used in the control group. Our study was approved by the institutional review board of the hospital and was conducted in accordance with the ethical principles. Written informed consent was obtained from each participant.

#### 2.1.1. Inclusion Criteria

Inclusion criteria are as follows: (1) aged 18-60 years, unilateral fresh closed calcaneal fracture; (2) calcaneal fractures consistent with Sanders II, III; and (3) complete relevant examinations before surgery, no obvious contraindications, and informed consent of patients.

#### 2.1.2. Exclusion Criteria

Exclusion criteria are as follows: (1) pathological fracture or old fracture and open fracture, (2) patients complicated with malignant tumor, (3) patients with acute cardiovascular and cerebrovascular diseases, (4) patients with diabetes, and (5) having varicose veins in the lower extremities.

## 3. Research Methods

### 3.1. Preoperative Preparation

Complete the laboratory examination and assess the patient's general condition after admission. After routine preoperative examination, the affected foot was raised with an elevating pad, local cold compress, and intravenous infusion of mannitol to reduce swelling. After a positive skin fold test, the operation was prepared. Acetaminophen tramadol was taken orally during this period.

CT thin layer scanning was performed on the calcaneal bone and contralateral normal calcaneal bone in the experimental group and control group. At the same time, the preplastic plate of the subtalar joint applied in the tarsal sinus approach and the anatomical locking plate applied in the L-shaped incision approach were scanned by a CT thin layer (Figure 1), and the data results were stored in DCM format files. The data of healthy calcaneus was imported into the 3D reconstruction software Mimics 21.0.

Threshold segmentation, region growth, 3D modeling, and other techniques were used to reconstruct a 3D bone model and generate a calcaneus model. After smoothing, 3D simulated images of the calcaneus with symmetry to the healthy side were generated by mirror technology, and the corresponding calcaneus model was generated by 3D printing technology, which was used as the standard of reduction of the affected side (Figure 2).

CT data of affected calcaneus were imported into Mimics 21.0 software. Major calcaneal fractures were marked using the calcaneal model generated after the unitary side image as the standard. Simulated fracture reduction in Mimics software can provide prospective guidance for intraoperative fracture reduction intuitively.

Boolean operation technique was used to fuse the plate and screw to generate the prototype of the navigation template. After appropriately trimming the shape of the navigation template and generating the STL format file, 3D printing equipment was used to make the model of reduced heel bone fracture on the affected side and the navigation template model was used for preoperative use after disinfection (Figure 3).

### 3.2. Surgical Methods

All surgeries were performed by associate chief physicians with similar surgical skills in the First Affiliated Hospital of Henan University of Science and Technology. The operation time was less than 3 hours, and one group of cefuroxime was routinely used preoperatively to prevent infection. After endotracheal intubation under general anesthesia+B ultrasound-guided nerve block anesthesia, the patient was placed in a lateral decubitus position. After the pressure tourniquet was fixed, the pressure was adjusted to 500 mmHg and the tourniquet was released every 90 minutes for 15 minutes. Routine disinfection and towel spreading were done.

#### 3.2.1. Tarsal Sinus Approach

The incision was made from 1 cm below the tip of the lateral malleolus to the base of the fourth metatarsal bone (Figure 4), and the incision length was appropriately extended according to the intraoperative needs (Figure 5). The isometric surface of the calcaneocuboid joint was exposed by incising the skin and subcutaneous fascia (Figure 6). The width, height, and varus deformity of the subtalar articular surface and calcaneus were restored, and temporary fixation with Kirschner wire was performed longitudinally on the posterior side of calcaneus tubercles. After satisfactory reduction effect was observed under the perspective, the preformed subtalar joint plate, which had been disinfected before surgery after simulated reduction, was placed in the position of the subtalar joint on the lateral wall of the calcaneus. After Kirschner wire adjustment, the screw was driven into the calcaneus according to the preset nail path (Figure 7). The second fluoroscopy proved that the reduction effect was satisfactory, and the traction Kirschner wire was removed. A large amount of normal saline was rinsed, a negative pressure drainage ball was indignant, the incision was closed layer by layer, and sterile auxiliary materials were wrapped up after disinfection.

#### 3.2.2. L-Shaped Incision Approach

From about 4 cm above the lateral malleolus at the front edge of the Achilles tendon, down to the dorsus and plantar skin junction, and then make arc fold forward, direct to the base of the fifth metatarsal near the side (Figure 8). Carefully separate the periosteum and superficial soft tissue and lift them upward at the depth of the peroneal longus tendon sheath (Figure 9). Three Kirschner wires were inserted into the cuboid, talus and lateral malleolus, respectively, to support the full-layer flap. Free the peroneus tendon to expose the subtalar articular surface as fully as possible. The Kirschner wire was inserted according to the preoperative deductive model. Combined with periosteal stripper and Kirschner wire, traction and pry reduction were performed to restore the calcaneal Böhler Angle, Gissane Angle, calcaneal width, height and varus deformity. After satisfactory reduction of the calcaneus shape and subtalar articular surface, the calcaneus navigation template was taken to test its fit with the external wall of the calcaneus. After adjusting the fast position of calcaneus fracture, the Kirschner wire was inserted into the preset needle path (Figure 10). After satisfactory reduction was determined by fluoroscopy, the defect site was enriched with allograft according to preoperative expectations to support the articular surface and maintain the shape of the calcaneus (Figure 11). Then, the navigation template was removed, and the preplastic anatomical plate was inserted and attached to the lateral wall of the calcaneus. The screw fixation plate was drilled in according to the preset nail path position before surgery (Figure 12). The second fluoroscopy proved that after good reduction and fixation, the incision was repeatedly washed with a large amount of normal saline, and a negative pressure drainage ball was indignant. The incision was sutured layer by layer, and sterile dressing was wrapped.

### 3.3. Postoperative Management

The negative pressure drainage ball was removed when the drainage flow was less than 50 ml within 24-48 h after surgery. Routine postoperative use of tranexamic acid for 1 day, oral administration of 1 tablet of acetaminophen tramadol/time, 3 times/day, elevation of the affected limb, and active application of drug-assisted detumescence. After surgery, anteropositive and lateral X-rays of the affected foot were routinely taken, and the patients were instructed by the same personnel to do functional exercises. Reexamination was performed at 1, 3, 6, and 12 months after discharge. After fracture healing, X-ray examination was performed every six months. Outpatient follow-up was performed to record functional recovery.

### 3.4. Observation Indicators

Preoperative and postoperative calcaneal width [16], calcaneal length [17], Böhler angle, Gissane angle, reduction of subtalar articular surface, operative time, hospital stay, operative duration, intraoperative blood loss, and postoperative fracture healing time were collected and measured.

Functional assessment was performed using the Maryland Foot sScore (MFS) system. The total score of the system is 100 points, which is divided into function and pain, accounting for 55 points and 45 points, respectively. The assessment included walking distance, gait, stability, walking AIDS, footwear, ground requirements for walking, ascending stairs, and walking, appearance, and mobility. A score of 90-100 is excellent, 75-89 is good, 50-74 is medium, and <50 is poor.

### 3.5. Statistical Methods

In this study, SPSS 24.0 statistical software was used to classify and sort out the data collected before, during and after surgery, and conduct statistical operation processing and analysis. Normal distribution analysis was carried out on the measurement data. If the data met the normal distribution, *t*-test was adopted; if not, nonparametric rank sum test was adopted. Chi-square test was used for counting data, and *P* < 0.05 indicated statistically significant difference.

## 4. Results

### 4.1. General Information

After inclusion of exclusion criteria, 40 postoperative patients were selected for comparison of preoperative and postoperative general data and preoperative and postoperative fracture-related indicators. Statistical software was used for analysis and processing to obtain relevant tables.

There were no significant differences in gender, age, Sanders classification, and affected limbs between 2 groups (*P* > 0.05). It can be considered that the case data of the two groups are basically the same and comparable, see Table 1.

### 4.2. Comparison of Preoperative and Postoperative Imaging Data

There were no significant differences in preoperative and postoperative calcaneal width, height, Böhler angle, and Gissane angle between 2 groups (*P* > 0.05). It showed that there is no significant difference between the experimental group and the control group in the comparison of the above imaging data.

There was no significant difference in the reduction of the subtalar articular surface before surgery (the subtalar articular surface displaced of control group is 16, and experimental group is 18), but there was statistical significance between the experimental group and the control group after surgery (the subtalar articular surface displaced of the control group is 4, and the experimental group is 1). This indicates that the experimental group, namely, the tarsal sinus approach, is superior to the control group, namely, the lateral L-shaped incision approach for the reduction of the subtalar articular surface, see Table 2.

### 4.3. Postoperative Functional Score

In postoperative follow-up, the total MSF score of the experimental group (91.36 ± 2.58) and the control group (90.12 ± 4.85) showed no significant difference between the two groups in functional recovery (Table 3).

### 4.4. Complications

Postoperative complications in the two groups were 5 cases (25%) in the experimental group and 1 case (5%) in the control group, the difference was statistically significant (*t* = 11.451, *P* < 0.001). The results showed that the incidence of postoperative complications was significantly lower with the tarsal sinus approach than with the lateral L-incision approach (Table 4).

## 5. Discussion

In the past century, a variety of treatments for displaced calcaneal fractures have been proposed, ranging from closed reduction to indirect reduction, limited open reduction to open reduction, but no clear consensus has been formed [18]. In recent years, with the development of digital computers and the application of 3D printing technology in orthopedics, comprehensive, fine, precise, and personalized treatment of calcaneal fracture has made great progress, and the previous problems of calcaneal defect and necrosis have been well solved [19].

The surgical treatment of calcaneal fracture has been developed in a variety of ways, and three approaches have been recognized by surgeons, including the lateral L-shaped incision approach, the tarsal sinus approach (STA), and the percutaneous approach.

The lateral extension incision was first proposed by Zwipp and colleagues in 1989 [5]. During the operation, a question about whether bone grafting is necessary for bone defects after reduction of severe calcaneal collapse was raised. According to 3D printing technology, the cancellous bone inside the calcaneal bone was simulated before reduction after compression, and a certain amount of allograft bone could be filled to maintain the integrity and supporting characteristics of the calcaneal bone. It provides anatomic location for strong internal fixation of plates and screws and restores the stability of the Böhler angle [20].

The tarsal sinus approach can enter the subtalar joints and at the same time with roll joints and calcaneal thrust forward [20]. In this study, the tarsal sinus minimally invasive approach was used in the experimental group and the results showed that compared with the lateral L incision, the L incision approach is relatively large, perioperative blood loss, and tarsal sinus minimally invasive. Compared with 98.77 cases of 18.65 ml in the control group and 89.56 + 17.54 ml in the experimental group (*P* > 0.05), the blood loss between the two groups was not statistically significant. The reason for this result was that, on the one hand, we performed pneumatic tourniquet in the patient's groin before surgery for intraoperative hemostasis. The operation time of both groups was completed within the time of setting a pneumatic tourniquet (90 minutes). Tourniquet intervention may significantly control the amount of blood loss in the incision, so that there is no significant difference between the two. On the other hand, the application of 3D printing technology, thorough preoperative surgical planning and deduction, and the application of navigation template for strong internal fixation can greatly shorten the operation time, so that the amount of blood loss can be significantly controlled. In addition, the intraoperative weighing of hemostatic gauze and collection of flushing fluid may also lead to deviation of experimental results.

The operation time of tarsal sinus approach is generally short. Therefore, soft tissue conditions, especially swelling, have relatively little influence on wound healing.

Compared with the results of postoperative soft tissue complications, the incidence of incision infection and skin edge necrosis was significantly higher with the L-shaped incision approach compared with the tarsal sinus approach, which was basically consistent with the results of related studies [21, 22]. However, it is certain that the intervention of 3D printing technology can significantly shorten the operation time, remove the pressure of the surrounding soft tissue caused by the fracture deformity, and restore the blood supply of the affected limb as soon as possible.

If the sural nerve is not clearly identified or the sural nerve is overstretched during the operation, the sural nerve is vulnerable to injury. In this study, one patient was found to feel slight numbness and discomfort in the lateral wall during the follow-up, which was considered to be caused by extrusion of sural nerve by screw or plate. The symptoms disappeared after internal fixation one year after surgery. With 3D printing technology, detailed preoperative deduction, fracture reduction, and navigation-template-assisted internal fixation can effectively shorten the operation time and significantly reduce the incidence of postoperative wound complications. Of course, the sample size of this study is limited, which may lead to some deviations in the results.

For displaced calcaneal intra-articular fractures, nonsurgical treatment and improper reduction or fixation often result in painful malunion or nonunion with severe functional deficits [23]. This study found that no malunion of fracture occurred in the two groups of patients assisted by 3D printing technology. Therefore, it is not difficult to see that the personalized and accurate application of 3D printing technology in fracture surgery can effectively reduce the occurrence of malunion.

Although 3D printing technology has many advantages in the application of preoperative surgical method formulation and instruction, there are still some limitations that need to overcome. First of all, the 3D printing auxiliary technology we used is only based on the bone CT model, so the information expression of adjacent soft tissues and blood vessels is not good. In addition, there is a certain time lag between the fracture data from CT scan and the output of fracture physical model, so it lacks timeliness for emergency surgical cases. In addition, for patients with severe comminuted fractures, current 3D printing technology cannot distinguish between the smallest fracture fragments. We have not applied 3D printing technology in postoperative rehabilitation, so the research on postoperative rehabilitation and functional exercise needs to be further explored. I believe that in the near future, 3D printing technology will certainly break through the bottleneck and leave a mark in the history of human medicine.

## 6. Conclusion

The experimental group was compared with the control group based on 3D printing technology, and it was found that the experimental group was significantly better than the control group in terms of operation time, intraoperative fluoroscopy times, and success rate of reduction of subtalar articular surface. The incidence of postoperative complications and the recovery of postoperative foot function and MSF score of foot function were better than the control group, but there was no significant difference. Combined with 3D printing technology, it has obvious advantages in shortening the operative time, precise reduction of fracture block, and reduction of secondary trauma during surgery and is conducive to the functional recovery of the affected foot after surgery.

## Figures and Tables

**Figure 1:** Steel plate model.

**Figure 2:** Reduction of the fracture was performed on the affected side based on the mirror image of the healthy side.

**Figure 3:** (a) The navigation template L-shaped incision navigation template and (b) tarsal sinus approach navigation template.

**Figure 4:** Tarsal sinus approach incision.

**Figure 5:** Calcaneocuboid joints are exposed.

**Figure 6:** Kirschner wire longitudinal fixation.

**Figure 7:** Restore subtalar articular surface leveling.

**Figure 8:** L-shaped incision approach.

**Figure 9:** Separate the lateral soft tissue of the calcaneus.

**Figure 10:** Fixed navigation template.

**Figure 11:** Good position of reduction confirmed after fluoroscopy.

**Figure 12:** Internal fixation with preplastic anatomic plate.

**Table 1:** Comparison of general conditions between the two groups.

	Control group	Experimental group	*T* value	*P* value
Gender (male/female)	16/4	18/2	2.862	0.090
Age (years old)	38.26 ± 11.18	37.80 ± 14.29	0.113	0.910
Preoperative detumescence time (d)	8.13 ± 3.50	9.24 ± 2.31	1.183	0.244
Sanders classification (II/III)	15/5	14/6	0.457	0.498
Affected side (right/left)	14/6	15/5	0.457	0.498
Duration of antibiotic use (d)	5.53 ± 3.24	5.48 ± 4.18	0.042	0.966
Operation time (min)	70.52 ± 13.16	55.24 ± 12.25	3.800	<0.001
Peroperative bleeding (ml)	98.77 ± 18.65	89.56 ± 17.54	1.608	0.119
Number of perspectives	6.56 ± 1.72	3.88 ± 1.05	5.947	<0.001
Fracture healing time (months)	3.24 ± 0.52	3.08 ± 0.58	0.918	0.364

**Table 2:** Comparison of imaging indicators between the two groups before and after surgery.

Type		Control group	Experimental group	*T* value	*P* value
Calcaneal width (cm)	Preoperative	43.25 ± 1.87	44.08 ± 2.85	1.088	0.283
	Postoperative	32.85 ± 2.38	34.14 ± 3.06	1.488	0.145
Calcaneal height (cm)	Preoperative	35.05 ± 1.82	33.95 ± 3.01	1.398	0.170
	Postoperative	41.89 ± 2.56	42.44 ± 2.82	0.645	0.522
Böhler angle	Preoperative	16.18 ± 3.06	16.04 ± 2.75	0.152	0.879
	Postoperative	28.31 ± 3.14	29.24 ± 2.76	0.994	0.326
Gissane angle	Preoperative	87.15 ± 3.36	88.81 ± 2.51	1.770	0.084
	Postoperative	130.98 ± 3.52	129.25 ± 2.87	1.703	0.096

**Table 3:** Postoperative MSF foot function scores of the two groups.

	Control group	Experimental group	*T* value	*P* value
Pain	43.24 ± 2.21	43.33 ± 1.50	0.151	0.881
Function	33.62 ± 2.46	34.33 ± 1.21	1.158	0.254
Appearance	5.26 ± 0.75	4.85 ± 0.78	1.694	0.098
Range of motion	4.12 ± 0.74	3.75 ± 0.55	1.795	0.081
MSF	90.12 ± 4.85	91.36 ± 2.58	1.001	0.319

**Table 4:** Comparison of postoperative complications between the two groups.

	Control group	Experimental group	*T* value	*P* value
Number	20	20		
Infection	1	0	1.025	0.311
Subtalar arthritis	1	0	1.025	0.311
Flap edge necrosis	2	1	0.360	0.548
Sural nerve injury	1	0	1.025	0.311
Sum total	5 (25%)	1 (5%)	11.451	<0.001

## Data Availability

The data used to support this study is available from the corresponding author upon request.
